# Effects of Voltage-Gated K^+^ Channel on Cell Proliferation in Multiple Myeloma

**DOI:** 10.1155/2014/785140

**Published:** 2014-06-08

**Authors:** Wei Wang, Yuying Fan, Shuye Wang, Lianjie Wang, Wanting He, Qiu Zhang, Xiaoxia Li

**Affiliations:** ^1^Department of Hematology, The First Affiliated Hospital of Harbin Medical University, 23 Youzheng Street, Nangang District, Harbin 150001, China; ^2^The Second Affiliated Hospital of Harbin Medical University, College of Nursing, Harbin 150086, China

## Abstract

*Objective*. To study the effects and underlying mechanisms of voltage-gated K^+^ channels on the proliferation of multiple myeloma cells. *Methods*. RPMI-8226 MM cell line was used for the experiments. Voltage-gated K^+^ currents and the resting potential were recorded by whole-cell patch-clamp technique. RT-PCR detected Kv channel mRNA expression. Cell viability was analyzed with MTT assay. Cell counting system was employed to monitor cell proliferation. DNA contents and cell volume were analyzed by flow cytometry. *Results*. Currents recorded in RPMI-8226 cells were confirmed to be voltage-gated K^+^ channels. A high level of Kv1.3 mRNA was detected but no Kv3.1 mRNA was detected in RPMI-8226 cells. Voltage-gated K^+^ channel blocker 4-aminopyridine (4-AP) (2 mM) depolarized the resting potential from −42 ± 1.7 mV to −31.8 ± 2.8 mV (*P* < 0.01). The results of MTT assay showed that there was no significant cytotoxicity to RPMI-8226 cells when the 4-AP concentration was lower than 4 mM. 4-AP arrested cell cycle in G0/G1 phase. Cells were synchronized at the G1/S boundary by treatment of aphidicolin and released from the blockage by replacing the medium with normal culture medium or with culture medium containing 2 mM 4-AP. 4-AP produced no significant inhibitory effect on cell cycle compared with control cells (*P* > 0.05). *Conclusions*. In RPMI-8226, voltage-gated K^+^ channels are involved in proliferation and cell cycle progression its influence on the resting potential and cell volume may be responsible for this process; the inhibitory effect of the voltage-gated K^+^ channel blocker on RPMI-8226 cell proliferation is a phase-specific event.

## 1. Introduction

Multiple myeloma (MM) is the malignant proliferation of plasma cells involving more than 10 percent of the bone marrow. The multiple myeloma cell produces monoclonal immunoglobulins that may be identified on serum or urine protein electrophoresis. MM comprises about 1% of all cancers but more than 10% of all hematooncological diseases. Cytogenetic analysis of MM cells shows frequent mutations and chromosomal aberrations. There are reciprocal chromosomal translocations involving the IgH locus, chromosome 13 monosomy, loss of short arm of chromosome 17 and gains of the long arm of chromosome 1, and others. Chemotherapy with melphalan-prednisone is the standard regimen for multiple myeloma. Other treatment modalities include polychemotherapy and bone marrow transplantation. But only 50 to 60 percent of patients respond to these therapies. The aggregate median survival for all stages of multiple myeloma is three years.

Membrane ion channels are essential for maintaining cellular homeostasis and signaling. Thus, they contribute to the control of essential parameters such as cell volume, intracellular pH, and intracellular Ca^2+^ concentration. K^+^ selective ion channels form the largest ion channel protein family, which may be subdivided into voltage-gated and Ca^2+^-dependent K^+^ channels and so on. Evidence is growing that K^+^ channels play a central role in the development and growth of human cancer like those of prostate, colon, lung, breast, and others. In nonexcitable cells voltage-gated K^+^ channels (Kv) play a critical role in cell development, volume regulation, membrane potential maintaining, and cell proliferation [1, 2]. Lots of researches speculated that Kv channels are correlated with the initial event of T and B lymphocyte activation [3, 4]. In the present study, the existence of Kv on the MM cells was directly detected; the relation between the channel and cell proliferation, cell cycle, and cell volume was further investigated, and the underlying mechanism was also explored.

## 2. Materials and Methods

### 2.1. Cell Culture

The RPMI-8226 human multiple myeloma cell lines (gift from Professor Chen Zi-xing, Hematology Institute, Suzhou) were cultured with RPMI-1640 with glutamine (GIBCO) supplemented with 10% (v/v) fetal bovine serum (GIBCO) and 1% (w/v) penicillin/streptomycin in a humidified 5% CO_2_ incubator (Thermo) at 37°C. RPMI-8226 cells were counted by automatic cell counting system to assay the proliferation.

1 mL of bone marrow sample was collected from young adult donor using a needle, which was immediately transferred into a sterile tube containing 1% heparin solution. To isolate bone marrow mononuclear cells, the samples were centrifuged in a 1.077 g/mL Ficoll density gradient for 30 min. The cells in the white middle layer were isolated and resuspended in culture medium with DMEM (GIBCO) containing 10% (v/v) fetal bovine serum (GIBCO) and 1% (w/v) penicillin/streptomycin. Then 1 × 10^6^ cells were seeded in a 100 mm dish that was precoated with 0.1% gelatin and incubated at 37°C with 5% CO_2_ at 100% humidity. After 3 days, the medium containing floating cells was removed and new medium was added to the remaining adherent cells. These adherent cells were considered to be BMSCs. The medium was changed every 3 days. The third passages were used for the following experiments [5, 6].

### 2.2. MTT Assay

The MTT solution was added to each well (1.2 mg/mL) and incubation was done for 4 h. The absorbance value (*A*) was measured at 570 nm using a multiwell spectrophotometer (Mapada, China). The percentage of cell viability was calculated using the following formula: cell viability (%) =* A* of experiment well/*A* of control well × 100%.

### 2.3. Patch-Clamp Recording

For patch-clamp experiments, the cells were plated on cover glass which had been pretreated with 1 mg/mL poly-L-lysine. Then cells were transferred to a recording chamber which was attached on the stage of an inverted phase-contrast microscope. The microscope was coupled to a video camera system with magnification up to 1500x in order to monitor cell size during the experiments. Cells were bathed at room temperature (20–25°C) and then superfused by gravity at a rate of about 2–4 mL/min (bath volume 2 mL) with normal Tyrode's solution. The patch pipettes were made from Kimax capillary tubes (Vineland, NJ) using a vertical two-step electrode puller (Narishige PB-7, Japan) and the tips were fire-polished with a microforge (Narishige MF-83, Japan). The resistance of the patch pipettes was 3–5 MΩ when it was immersed in normal Tyrode's solution. Voltage-clamp potentials of step or ramp depolarization were generated by a programmable stimulator (Biologic SMP-311, France). Ionic currents were recorded in whole-cell clamp conditions with the use of a patch-clamp amplifier (Biologic RK-400, France) and amplified with a low-pass filter at 1–3 KHz. All potentials were corrected for liquid junction potential which developed at the tip of the pipette when the composition of pipette solution was different from that of bath. Tested drugs were applied by perfusion to the bath to obtain the final concentrations indicated.

Whole-cell voltage-clamp recordings were performed to record the voltage-dependent potassium currents in RPMI-8226 cells. Axopatch 200B patch-clamp magnifying instrument is controlled by the computer. The recording pipette was pulled using borosilicate capillaries. The resistance of the pipette was 3–5 MΩ when it was filled with the pipette solution. All recordings were done at room temperature (21°C). The internal solution contained (mM) K-aspartate 135, MgCl_2_ 2, EGTA 1.1, CaCl_2_ 0.1, and HEPES-KOH buffering liquid 10, adjusted to pH 7.2 with 1 M KOH (280–300 mOsm). The electrode external solution contained (mmol/L) NaCl 136.5, KCl 5.4, CaCl_2_ 1.8, MgCl_2_ 0.53, glucose 5.5, and HEPES-NaCl buffering liquid 5, adjusted to pH 7.2 with 1 M NaOH (280–300 mOsm). For the voltage-dependent potassium currents recording, the membrane voltage was stepped to −90 mV for 1 s followed by a ramp to +50 mV. All the records are kept in the hard disk for the postexperiment analysis.

### 2.4. RT-PCR Assay

RNA was extracted from RPMI-8226 cells using Trizol reagent (Invitrogen) according to the manufacturer's instructions. Two micrograms of RNA was reverse-transcribed and the products were amplified with cDNA-specific primers (Roche). The sequence of primers (Jinsite Biotechnology) for RT-PCR was as follows: Kv1.3 forward: 5′-TCGCCATCGTGTCCGT-3′ and reverse: 5′-CCATTGCCCTGTCGTT-3′; Kv3.1 forward: 5′-GAGGACGAGCTGGAGATGAC-3′ and reverse: 5′-GGCAGAAGATGACACGCATG-3′; *β*-actin forward: 5′-AGCGGGAAATCGTGCGTG-3′ and reverse: 5′-CAGGGTACATGGTGGTGCC-3′. The PCR was performed with 40 cycles of denaturation at 95°C for 30 seconds, annealing at 60°C for 30 seconds, and extention at 72°C for 60 seconds, with an initial denaturation at 95°C for 10 minutes and a final extension at 72°C for 7 minutes. *β*-Actin served as control. The experiments were repeated twice. The PCR product was loaded onto 2% agarose gel for electrophoresis and visualized using Gel Doc XR imaging system (Bio-Rad).

### 2.5. Cell Cycle and Cell Volume Analysis

RPMI-8226 cells (1.0 × 10^6^ cells) were washed twice with PBS and then fixed with 70% ice-cold ethanol for 24 hours at 4°C. After being washed with PBS one more time, fixed cells were incubated with Tris-HCl buffer (pH 7.4) containing 10 *μ*g/mL RNA enzyme for 30 min at 37°C. The cells were stained with propidium iodide (Becton-Dickinson). The distribution of nuclear DNA contents was analyzed by flow cytometry (FACS Calibur, Becton-Dickinson). Data were collected using CellQuest software and analyzed by ModFit LT software version 2.0.

RPMI-8226 cells (1.0 × 10^6^ cells) were washed twice with PBS and resuspended in 1 mL PBS. Cells were detected with a flow cytometer. Ten thousand events were collected and the data was analyzed with CellQuest software. Forward side scatter (FSC) describing cell size was used to measure the cell volume [7].

### 2.6. Statistical Analysis

Current inhibition rate was calculated using the following formula: (|*I*_control_| − |*I*_measure_|)/|*I*_measure_|. Data values are presented as means ± SDs. Student's paired *t*-test was used to analyze the difference between the control and 4-AP-treated cells. All *P* values <0.05 were considered to be significant.

## 3. Results

### 3.1. Detection of Kv on MM Cells

To study the effect of voltage-gated potassium channels on multiple myeloma cell proliferation, we first measured whether the currents were voltage-gated potassium currents. The mean resting potential and cell capacitance were −42 ± 2 mV and 37.5 ± 2 pF, respectively (*n* = 40). Membrane currents were evoked at 0.1 Hz by various step pulses with a duration of 1 s before and after the addition of 4-AP. Under controlled conditions, when the cell was held at −80 mV, the depolarizing pulses which are more than −30 mV can elicit the outward currents. The amplitudes of these currents were increased with greater depolarization pulses. When the cells were held at −80 mV, the measured potentials were −54 ± 1 mV, −49 ± 3 mV, −30 ± 1 mV, and −10 ± 2 mV (*n* = 11) according to extracellular K^+^ concentrations of 5.4 mM, 10 mM, 40 mM, and 80 mM. These results indicate the changes of membrane currents dependence on the extracellular K^+^ concentration. Furthermore the elicited current was voltage-gated and could be deactivated by repeated depolarization.

### 3.2. Kv Channels Subtype Expression in RPMI-8226 Cells

There are two kinds of Kv channels expressed in the lymphocytes, n-type and l-type, and they are coded by Kv1.3 and Kv3.1 genes, respectively [8]. As multiple myeloma cells originate from pre-B lymphocytes, we assayed the mRNA expression of the two channels in RPMI-8226 cells by RT-PCR. A high level of Kv1.3 mRNA was detected and no Kv3.1 mRNA was detected (Figure 1), which indicated that the n-type Kv channels exist in RPMI-8226 cells.

### 3.3. Effects of 4-AP on Resting Membrane Potential in RPMI-8226 Cells

Under whole-cell current-clamp conditions, 5 minutes being held, 4-AP (2 mM) depolarized the resting potential from −42 ± 1.7 mV to −31.8 ± 2.8 mV (*n* = 6, *P* < 0.01). This result demonstrated that Kv channels play an important role in maintaining cell membrane potential.

### 3.4. Effects of 4-AP on Current-Voltage (*I-V*) Relation of K^+^ Channels in RPMI-8226 Cells

Original records from a typical cell before and after addition of 2 and 10 mM 4-AP are shown in Figure 2(a). After 4-AP was removed, Ikv could not return completely to the control level. The current-voltage relations in the absence and presence of 4-AP (2 mM/10 mM) were shown in Figure 2(b). The effect of 4-AP on the current-voltage relations in the range of −90 mV and +50 mV was demonstrated in 6 RPMI-8226 cells. At +50 mV, 4-AP (2 mM/10 mM) reduced the peak amplitudes of Ikv by 48.2 ± 3.45% and 82.8 ± 7.45%, respectively, compared to the control.

### 3.5. Effect of 4-AP on RPMI-8226 Cell Proliferation and Cell Cycle

Cytotoxicity of 4-AP to RPMI-8226 cells was studied by applying different concentrations of 4-AP in the normal culture medium for up to 4 days. Viability of control and 4-AP-treated cells was determined by MTT assay. When 4-AP concentration was less than 4 mM, no significant cytotoxicity to RPMI-8226 cells was observed (Figure 3(a)).

The effect of 4-AP on RPMI-8226 cell proliferation was evaluated by counting cell numbers. Introduction of 2 mM 4-AP, a dose similar to that used by other groups [9], for 48 h caused a significant decrease in RPMI-8226 cell number (Figure 3(b)). A dose-response curve for 4-AP inhibition of cell proliferation was obtained (Figure 3(c)). In bone marrow stromal cells and RPMI-8226 cells, the calculated half-maximal inhibitory concentration of 4-AP was 6.1 ± 0.2 mM and 4.4 ± 0.3 mM separately (*P* < 0.05), respectively, demonstrating higher sensitivity of MM cells to 4-AP.

The effect of 4-AP on cell cycle was also evaluated. RPMI-8226 cells were cultured in the normal medium, serum-deprived medium, or medium containing 2 mM 4-AP for 24 h and then collected for cell cycle analysis using flow cytometry. The cells in G0/G1 phase were increased from 32.5 ± 4% in control group (cultured in the normal medium) to 61.5 ± 4.7 and 78.9 ± 4.0% in serum-deprived group and 4-AP- (2 mM) treated group, respectively (Figure 4). S phase population significantly decreased from 60.6 ± 6.1% in control group to 35.6 ± 4.4% in 4-AP-treated group (Figure 4).

To determine the phase-specific blockage of 4-AP in cell cycle, RPMI-8226 cells were synchronized at the G1/S boundary by application of aphidicolin, a DNA polymerase inhibitor. After incubation for 16 h with 5 mg/mL aphidicolin, RPMI-8226 cells passed the G1 checkpoint at the end of the G1 phase and approached the beginning of the S phase. The cells were then released from blockage by replacing the medium with normal culture medium (control group) or medium containing 2 mM 4-AP. However, 4-AP did not inhibit cell cycle progression that passed G1 checkpoint, indicating that 4-AP specifically inhibited G1 phase which requires the involvement of K^+^ channel for cell proliferation (Table 1).

### 3.6. Effect of 4-AP on RPMI-8226 Cell Volume

It has been shown that alterations of cell volume can affect intracellular signaling pathways (26). We examined the effect of inhibition of K^+^ channel activity by 4-AP on cell volume (see Figure 5 and Table 2). Cell volume is in direct proportion to the intensity of forward side scatter (FSC), which is used to measure the cell volume [7]. RPMI-8226 cells were cultured in the presence of 2 mM 4-AP for 24 h. The suppression of K^+^ channel activity resulted in 12 ± 3.2%, 19.3 ± 1.6%, and 28 ± 4.3% (*n* = 3) increase in cell volume compared with control cells, respectively (Table 1). Our data are in agreement with the model proposed by Dubois and Rouzaire-Dubois [10], in which the K^+^ channel plays an important role in controlling cell volume.

## 4. Discussion

It has been reported that voltage-dependent potassium channel (Kv) is found in T lymphocytes, B lymphocytes, and other cells [8]. In this study, we noticed the presence of Kv channels, which is a type of K^+^ channels coded by Kv1.3 gene, in RPMI-8226 multiple myeloma cells. The currents exhibited the kinetic, voltage-dependent, and pharmacological characteristics as expected. As found in other preparations, the voltage-activated K^+^ currents were sensitive to 4-AP.

K^+^ channels' activity has been implicated in cellular proliferation in a variety of cell types [11]. Although 4-AP has previously been reported to inhibit the proliferation of tumor cells [12, 13], this is the first study to show such an effect in RPMI-8226 multiple myeloma cells.

In previous studies, K^+^ channel blockers were found to inhibit mitogenesis of various cell types, which suggested that K^+^ channels are required for cell proliferation and signal transduction in mitogenesis [3, 14]. The suppression of K^+^ channels' activity could weaken the immune system by inhibiting T lymphocytes proliferation. Accordingly, human Kv1.3 has been recognized as an excellent therapeutic target for modulating immune system [14]. However, it is unclear whether voltage-gated potassium channels in MM cells membrane are involved in cell proliferation.

In human T lymphocytes, voltage-gated K^+^ channels are crucial to transmembrane potential and cell proliferation in response to mitogenic stimulation [15, 16]. In our study 4-AP induced a significant decrease of membrane potential in a dose-dependent manner in MM cells. The effect of membrane potential variations under the control of K^+^ channels would be involved not only in regulating Ca^2+^ influx, which is well established as a crucial factor for cell proliferation, but also in maintaining the driving force for Na^+^-dependent nutrient transport and influencing the intracellular pH [17]. On the other hand, a large number of reports show that a transient hyperpolarization is required for the progression of the early G1 phase in cell cycles, and K^+^ channels activated by mitogenic signals mainly control the hyperpolarization [18]. Our data indicate that suppression of the K^+^ channels by 4-AP inhibits RPMI-8226 cells proliferation and results in accumulation of G1 phase cells. Arrest of RPMI-8226 cells at the G1/S boundary with aphidicolin revealed that RPMI-8226 cells that have progressed through the G1 checkpoint are capable of entering S phase and synthesizing DNA, independent of the presence of channel blocker. Our results support the hypothesis that inhibition of the K^+^ channels by 4-AP on RPMI-8226 cells proliferation is a phase-specific event. It is suggested that the mechanism of cell proliferation inhibition should be as follows: K^+^ channel blocker inhibits K^+^ flux, which leads to membrane potential depolarization and inhibition of transient hyperpolarization and therefore intracellular environment changes, such as the levels of Ca^2+^, Na^+^, and pH and the related enzymes' activation.

In addition to controlling membrane potential, plasma membrane K^+^ channels are also critical components in cell volume regulation [2]. Heterologous expression of Kvl.3 channels in mouse CTLL-2 cells, which were unable to control cell volume before gene transfection, reconstitutes their ability to regulate cell volume [2]. In the present study, we observed that RPMI-8226 cell volume increases up to 28 ± 4.3% after 24 h suppression of K^+^ channels by 4-AP. The volume increase may play a regulatory role in cell growth, either by altering intracellular ions concentration or by altering the activity of mitogen-activated kinases [19]. In fact, glioma cells show their highest proliferation rate within a relatively narrow range of cell volumes, with decreased proliferation both over and under that optimal range [20], namely, “cell size checkpoint,” which exists in many types of mammalian cells. The hypothesis brought forward by Dubois and Rouzaire-Dubois [10] postulates that K^+^ channels responsible for cell volume regulation have an admission function in cell proliferation through controlling volume in such a way that crucial solutes, including Na^+^ which is very important to DNA synthesis and the second messenger Ca^2+^, can maintain an appropriate concentration to support proliferation or activate mitogen-activated protein kinases (MAPKs). Thus the mechanism of cell volume regulation in proliferation needs to be further explored.

## 5. Conclusion

In conclusion, we have demonstrated that suppression of K^+^ channels' activity can markedly inhibit RPMI-8226 cell proliferation and arrest cells in G1 phase of cell cycle. Our results additionally support the notion that voltage-gated K^+^ channels contribute to control cell growth through the G1/S transition in the cell cycle. And further studies are required to investigate the mechanism of how the K^+^ channels mediate signals involved in cell growth.

## Figures and Tables

**Figure 1:** Detection of Kv1.3 and Kv3.1 transcription in RPMI-8226 cells by RT-PCR. M: molecular weight marker; 1: *β*-actin; 2: Kv3.1; 3: Kv1.3.

**Figure 2:** Effect of 4-AP on RPMI-8226 cells' voltage-gated potassium channel currents. (a) Current curve noted before and after 2 mM and 10 mM 4-AP treatment and 10 min washing. Stimulation procedure: currents were studied using a depolarizing pulse of 1 sec duration and 500 ms interval from −90 to +50 mV in 10 mV steps driven from a holding membrane potential of −80 mV. (b) Effect of 4-AP on voltage-current curve in RPMI-8226 cell line.

**Figure 3:** Effect of 4-AP on RPMI-8226 cell viability and cell proliferation. (a) Different concentrations of 4-AP ranging from 0.5 mM to 8 mM were added to examine viability in 24 h, 48 h, 72 h, and 96 h. Data were plotted as means ± SD. (b) Cells were divided and cultured in the normal medium, serum-free medium, and 2 mM 4-AP containing medium for 48 hours. (c) Effects of 4-AP in various concentrations on RPMI-8226 cells proliferation.

**Figure 4:** Effect of 4-AP of voltage-gated potassium channels blockage on cell cycle phases (*versus control, *P* < 0.05; **versus control, *P* < 0.01, *n* = 3).

**Figure 5:** Effect of 2 mM 4-AP on cell volume (100 times).

**Table 1:** Effect of 4-AP of voltage-gated potassium channels blockage on cell cycle phases.

	G0/G1	S	G2/M
Control group	52.42333	42.14	5.436667
4-AP 2 mM group	50.14667	43.73667	6.116667

**Table 2:** Effect of 2 mM 4-AP on cell volume at various time points.

Time	0 h	2 h	12 h	24 h
Intensity of FSC	320.3 ± 34.3	359.1 ± 34.4	382.0 ± 38.4	410.7 ± 51.1

## References

[1] Blackiston DJ, McLaughlin KA, Levin M (2009). Bioelectric controls of cell proliferation: ion channels, membrane voltage and the cell cycle. *Cell Cycle*.

[2] Bobak N, Bittner S, Andronic J (2011). Volume regulation of murine T lymphocytes relies on voltage-dependent and two-pore domain potassium channels. *Biochimica et Biophysica Acta—Biomembranes*.

[3] Yoo HY, Zheng H, Nam JH (2008). Facilitation of Ca^2+^-activated K^+^ channels (IKCa1) by mibefradil in B lymphocytes. *Pflugers Archiv European Journal of Physiology*.

[4] Beeton C, Barbaria J, Giraud P (2001). Selective blocking of voltage-gated K^+^ channels improves experimental autoimmune encephalomyelitis and inhibits T cell activation. *Journal of Immunology*.

[5] Ciapetti G, Ambrosio L, Marletta G, Baldini N, Giunti A (2006). Human bone marrow stromal cells: in vitro expansion and differentiation for bone engineering. *Biomaterials*.

[6] Ma N, Gai H, Mei J (2011). Bone marrow mesenchymal stem cells can differentiate into type II alveolar epithelial cells in vitro. *Cell Biology International*.

[7] Schuette WH, Shackney SE, Plowman FA, Tipton HW, Smith CA, MacCollum MA (1984). Design of flow chamber with electronic cell volume capability and light detection optics for multilaser flow cytometry. *Cytometry*.

[8] Grgic I, Wulff H, Eichler I, Flothmann C, Köhler R, Hoyer J (2009). Blockade of T-lymphocyte KCa3.1 and Kv1.3 channels as novel immunosuppression strategy to prevent kidney allograft rejection. *Transplantation Proceedings*.

[9] Woodfork KA, Wonderlin WF, Peterson VA, Strobl JS (1995). Inhibition of ATP-sensitive potassium channels causes reversible cell-cycle arrest of human breast cancer cells in tissue culture. *Journal of Cellular Physiology*.

[10] Dubois J-M, Rouzaire-Dubois B (1993). Role of potassium channels in mitogenesis. *Progress in Biophysics and Molecular Biology*.

[11] Wulff H, Castle NA, Pardo LA (2009). Voltage-gated potassium channels as therapeutic targets. *Nature Reviews Drug Discovery*.

[12] Cidad P, Jiménez-Pérez L, García-Arribas D (2012). Kv1.3 channels can modulate cell proliferation during phenotypic switch by an ion-flux independent mechanism. *Arteriosclerosis, Thrombosis, and Vascular Biology*.

[13] Jang SH, Choi SY, Ryu PD, Lee SY (2011). Anti-proliferative effect of Kv1.3 blockers in A549 human lung adenocarcinoma in vitro and in vivo. *European Journal of Pharmacology*.

[14] Lam J, Wulff H (2011). The lymphocyte potassium channels Kv1.3 and KCa3.1 as targets for immunosuppression. *Drug Development Research*.

[15] Leonard RJ, Garcia ML, Slaughter RS, Reuben JP (1992). Selective blockers of voltage-gated K^+^ channels depolarize human T lymphocytes: Mechanism of the antiproliferative effect of charybdotoxin. *Proceedings of the National Academy of Sciences of the United States of America*.

[16] Negulescu PA, Shastri N, Cahalan MD (1994). Intracellular calcium dependence of gene expression in single T lymphocytes. *Proceedings of the National Academy of Sciences of the United States of America*.

[17] Pardo LA (2004). Voltage-gated potassium channels in cell proliferation. *Physiology*.

[18] Kunzelmann K (2005). Ion channels and cancer. *Journal of Membrane Biology*.

[19] Matsuda S, Kawasaki H, Moriguchi T, Gotoh Y, Nishida E (1995). Activation of protein kinase cascades by osmotic shock. *The Journal of Biological Chemistry*.

[20] Rouzaire-Dubois B, Malo M, Milandri J-B, Dubois J-M (2004). Cell size-proliferation relationship in rat glioma cells. *GLIA*.

